# EERP-DPM: Energy Efficient Routing Protocol Using Dual Prediction Model for Healthcare Using IoT

**DOI:** 10.1155/2021/9988038

**Published:** 2021-05-06

**Authors:** Faris A. Almalki, Soufiene Ben Othman, Fahad A. Almalki, Hedi Sakli

**Affiliations:** ^1^Department of Computer Engineering, College of Computers and Information Technology, Taif University, P.O. Box 11099, Taif 21944, Saudi Arabia; ^2^PRINCE Laboratory Research, ISITcom, Hammam Sousse, University of Sousse, Sousse, Tunisia; ^3^College of Medicine, Majmaah University, Al Majma'ah, Saudi Arabia; ^4^MACS Research Laboratory, National Engineering School of Gabes, Gabes University, Gabes 6029, Tunisia; ^5^EITA Consulting 5 Rue du Chant des Oiseaux, Montesson 78360, France

## Abstract

Healthcare is one of the most promising domains for the application of Internet of Things- (IoT-) based technologies, where patients can use wearable or implanted medical sensors to measure medical parameters anywhere and anytime. The information collected by IoT devices can then be sent to the health care professionals, and physicians allow having a real-time access to patients' data. However, besides limited batteries lifetime and computational power, there is spatio-temporal correlation, where unnecessary transmission of these redundant data has a significant impact on reducing energy consumption and reducing battery lifetime. Thus, this paper aims to propose a routing protocol to enhance energy-efficiency, which in turn prolongs the sensor lifetime. The proposed work is based on Energy Efficient Routing Protocol using Dual Prediction Model (EERP-DPM) for Healthcare using IoT, where Dual-Prediction Mechanism is used to reduce data transmission between sensor nodes and medical server if predictions match the readings or if the data are considered critical if it goes beyond the upper/lower limits of defined thresholds. The proposed system was developed and tested using MATLAB software and a hardware platform called “MySignals HW V2.” Both simulation and experimental results confirm that the proposed EERP-DPM protocol has been observed to be extremely successful compared to other existing routing protocols not only in terms of energy consumption and network lifetime but also in terms of guaranteeing reliability, throughput, and end-to-end delay.

## 1. Introduction

The IoT is a new paradigm that is rapidly gaining ground in the modern wireless telecommunications applications. The basic idea behind this concept is the ubiquitous presence of a variety of things or objects around us such as Radio Frequency Identification (RFID), sensors, actuators, and cell phones. This happens through unique addressing schemes that enable nodes to interact with each other and cooperate with their neighbores to achieve common goals [1]. There are numerous IoT applications in many fields, such as smart buildings, industrial automation, medical aids, mobile health, smart education, assistance to the elderly, and intelligent energy management [2–8]. Moreover, research and development of employing intelligent sensors in medical field are vast, including home hospitalization, integration of microsensors in body, and emergency management [3].

In wireless sensors, the absence of restrictive electrical installations and the reduction of wire clutter connecting the sensors to the processing unit afford more liberty of movement for the patient [6]. Moreover, using IoT in the medical field offers many advantages and brings new comfort to patients such as patient mobility, remote monitoring of the elderly, and people with reduced mobility, efficient monitoring, monitor certain vital signs, enhanced quality of care, and long-term care [4, 5]. The healthcare using the IoT does not only improve the quality of life of patients, but also facilitate their real-time remote monitoring and the quick intervention in case of emergency (if the measurements reported by the sensors are abnormal) [7].

Medical sensors are characterized by small size, less storage, less processing capabilities, and energy constraint resources. These sensors are battery-powered, where frequent replacement of its battery is a sophisticated, costly and complicated medical procedure as some sensors get implanted inside the body, so surgical replacement is necessary [8–10]. In sequence, real-time monitoring of patients with sensors sending reliable medical information in regular bases requires extremely low power disruption [11].  Figure 1 shows typical structure of the healthcare surveillance system using IoT, where sensors are deployed in the human body to monitor parameters like temperature, heart rate, blood pressure, etc. These values can be read from the sensors and then get transmitted to the server, where physicians can access this data and evaluate it.

Motivated by the mentioned observations, and the upcoming related studies, this paper develops a novel Routing Protocol called “Energy Efficient Routing Protocol using Dual Prediction Model for Healthcare using IoT (EERP-DPM)” for Healthcare using the IoT that is designed to reduce the requirements of existing routing protocols, where the DPM is used to reduce transmissions between the sensor nodes and the medical server. This technique allows sensor nodes to avoid transmitting its sensed data to medical server if the predictions match the sensing data. Meanwhile, the medical server always presumes that its prediction reflects the real observation, unless it receives the data from the sensor node. The data is transmitted if it is different from the data predicted, where normal health data is forwarded to the Aggregator through deployed relay nodes. The data is considered critical if it is beyond the upper/lower limits of previously defined thresholds, where emergency data can be sent directly to the Aggregator. The proposed system was developed and tested using MATLAB software simulation, as well as being tested experimentally using MySignals HW V2 hardware platform. Both simulation and experimental results are compared to the E-HARP [12] and PCRP [13] protocols. The remainder of this paper is organized as follows: the related works are investigated in Section 2. Proposed network model design solution and goals are presented in Section 3, followed by the performance evaluation and discussion in Section 4. Finally, Section 5 concludes this paper.

## 2. Related Work

This section covers a survey of different approaches of routing protocols for IoT-based healthcare applications. Then, we used this review to highlight the research gaps and report our own research motivations by comparing it against existing works in the literature as presented in Table 1.

By knowing that sensors could consume about 70% energy on wireless communication with other nodes and/or with the server, solutions should be considered to work on this aspect [20]. Hence, routing protocols play vital role in providing effective communication between the sensors, to prolong the overall lifetime of networks via minimizing energy consumption that required forwarding data from sensor nodes to a medical-related server efficiently [21]. The traditional routing protocol is not a suitable solution for this type of network due to resource limitations [22], where, in the last decade, many works have been proposed by different researchers who focused on developing adaptive and robust routing protocols [10–27]. The various works use the congestion control techniques and maximizing battery efficiency to extend the network lifetime. However, several key issues stay as open challenges, where most researches did not widely focus on heterogeneity of healthcare data and deal with it [23].

The authors in [12] presented a routing scheme known as “Energy-Efficient Harvested-Aware Clustering and Cooperative Routing Protocol for Wireless Body Area Networks (E-HARP).” This scheme is a multiattribute-based harvested energy routing protocol, which takes different network-related parameters into consideration and selects an optimal forwarder node towards the sink node using two-phased technique. In the first phase, optimum CH is selected among the cluster members based on calculated Cost Factor (CF). The parameters used for calculation of CF are residual energy of SN, required transmission power, communication link signal-to-noise ratio (SNR), and total network energy loss. In the second phase, data are routed with cooperative effort of the SN, which saves the node energy by prohibiting the transmission of redundant data packets.

A Priority-based Congestion-avoidance Routing Protocol (PCRP) is proposed in [13], which is a technique that used IoT-based heterogeneous medical sensors for energy efficiency in healthcare wireless body area networks. Data criticality and QoS requirements are the prime importance of the proposed work. For normal data packet, the fitness function will be calculated based on three parameters, namely, signal-to-noise ratio (SNR), residual energy (RE), and node congestion level (NCL). SNR parameter is used for a better selection of path between sender and receiver. For highly important data, they have supposed a priority bit.

Researchers in [14] introduced a new routing protocol named “Green Communication for Wireless Body Area Networks: Energy Aware Link Efficient Routing Approach (ELR-W).” This protocol considers four parameters, residual energy, link efficiency, node to coordinator distance, and hop count, to construct a path cost model, which is used to select the next-hop node for transfer data. This cost function is subject to change with respect to parameters like hop count, link efficiency, and residual energy. The comparative performance evaluation has been carried out focusing on energy-oriented metrics under WBANs medical environments.

Ullah et al. in [15] proposed a complete novel scheme, which is proposed for WBANs, named as “Robust and Energy Harvested-aware Routing Protocol with Clustering Approach in Body Area Networks (EH-RCB).” The proposal is based on a system, in which tiny sensors nodes are placed on the human body to sense important health-related parameters and forward them to two sink nodes. It is designed to stabilize the operation of WBANs by choosing the best forwarder node, which is based on optimal calculated Cost Function (CF). The CF considers the link SNR, required transmission power, the distance between nodes, and total available energy (e.g., harvested energy and residual energy). To note, energy harvesting technique is adopted to provide additional energy to the sensor nodes in order to help out in prolonging the network lifetime.

The authors in [16] presented the “Energy Budget-based Multiple Attributes Decision Making Algorithm (EB-MADM),” which was designed to be low power and cluster-based routing mechanism. The algorithm selects an optimum node as cluster head, which has higher residual energy level and performs data routing at the cost of least network residual energy loss. EB-MADM selects a new cluster head for each transmission round and distributes cluster head load evenly among cluster nodes. Simulation results show better performance in terms of network stability, propagation delay, throughput, and network lifetime as compared to its counterparts.

Priority-based and energy-efficient routing for IoT systems (PriNergy) is considered in [17]. The proposed method is based on routing protocol for low power and lossy network (RPL) model, which determines routing through contents. Each network slot uses timing patterns when sending data to the destination, while considering network traffic, audio, and image data. In the proposed RPL model, if an error occurs in a parent member node, its members can remain alive until the convergence and configuration of the parentless parenthesis and their packets expire due to the time lapse.

Khan et al. [18] proposed the Energy Harvested and Cooperative Enabled Efficient Routing Protocol (EHCRP) for IoT-WBAN. The proposed protocol considers multiple parameters of WBANs for efficient routing such as residual energy of SNs, number of hops towards the sink, node congestion levels, Signal-to-Noise Ratio (SNR), and available network bandwidth. A path cost estimation function is calculated to select forwarder node using these parameters. Due to the efficient use of path-cost estimation process, the proposed mechanism achieves efficient and effective multihop routing of data and improves the reliability and efficiency of data transmission over the network.

Researchers in [19] proposed a protocol named Optimum Path Optimum Temperature Routing Protocol (OPOT). The proposed protocol maintains the temperature of node and communicates the sensed information to remote server with minimum delay and energy, thereby increasing the lifetime of sensor networks. It also considers the critical data signals to be sent when the temperature of node exceeds the admissible threshold limit. The obtained simulation results are compared with conventional routing protocols and analyzed that the proposed protocol has decreased delay, minimum energy, reduced power, uniform temperature distribution, and maximum lifetime of sensor node.

Motivated by the mentioned observations through the related studies, major portions that collected data from medical sensors are usually redundant, which means unnecessary transmission and, thus, high energy consumption. In this context, the reduction of transmission of such redundant data can be achieved using the proposed DPM. The idea of the proposed solution EERP-DPM runs a prediction model at both the sensing nodes and the base station to allow sensor nodes to avoid transmitting its sensed data to the base station, as long as the predictions match the readings. Meanwhile, the base station always presumes that its prediction reflects the real observation, unless it receives the corrections from the sensor node (since the sensor can compare the prediction with the real sensed measurement). The most essential benefit from the DPM is the ability to shrink traffic volume exchanged in the networks quite significantly. Besides, transmitting less data certainly saves sensor energy and, therefore, prolongs the lifetime of the entire network [12, 25–27].

To sum up, the proposed EERP-DPM system was developed and tested using MATLAB software simulation, besides hardware implementation using MySignals HW V2 platform, which is a noticeable and comprehensive contribution from the existing work in the literature. Moreover, the proposed solution runs a prediction model at both the sensing nodes and the base station to allow sensor nodes to avoid transmitting their sensed data to the base station, as long as the predictions match the readings. The medical server always presumes that its prediction reflects the real observation unless it receives the data from the sensor node. The data is transmitted if it is different from the data predicted, where normal health data are forwarded to the Aggregator through deployed relay nodes. The data is considered critical if it is beyond the upper/lower limits of previously defined thresholds, where emergency data can be sent directly to the Aggregator.

## 3. Proposed Design System and Architecture Model

This section contains system network architecture, followed by the proposed EERP-DPM solution.

### 3.1. System Network Architecture

The architecture considered in the proposed work is shown in Figure 2, where it can be utilized in a hospital and even locate remote patients. The architecture model of our proposed scheme comprises four architectural components: Medical Sensors Nodes, Relay Nodes, an Aggregator, and Medical Server.

- Medical Sensor Nodes: patients are equipped through wearable devices that form Wireless Medical Sensors (MSs). These heterogeneous sensors are either strategically implanted or placed on the body as wearable devices on human body to monitor body functions. Each sensor node is integrated with biosensors, which are body temperature, electromyography, electrocardiography, blood pressure, pulse-oximeter, and electroencephalography.
- Relay Nodes: patients are equipped through devices, named relay nodes, which can be easily replaced or recharged. The relay nodes reduce the transmitting distance between sensor nodes and Aggregator, where these nodes have two major advantages: (1) protecting the human tissues from heating effect and radiation and (2) decreasing energy consumption of sensor nodes during forwarding of sensing data. In this proposed solution, we placed three relay nodes, as discussed in Table 2.
- Aggregator: it is a special sensor node with a superior certain ability to calculate and communicate. Aggregation nodes, as the name suggests, will aggregate sensed data using aggregation functions. The patient's mobile device is used as the Aggregator. The Aggregator works as a router between the Medical Sensors nodes and the medical server. The placement of the Aggregator is at the centroid of placed sensor nodes. It uses different technologies such as cellular mobile networks (2G–5G) or WLANs for communication with medical server placed at distant location.
- Medical Server: it includes healthcare providers (e.g., doctors, physicians, nurses, and researchers). It possesses almost infinite storage capability and the computation of the resources. The server has the computation abilities to execute the calculations over the stored data including disease learning and prediction. On receiving the patient's health data, the doctor can get real-time situational awareness.

### 3.2. Proposed EERP-DPM Solution

In this subsection, we present the proposed solution of EERP-DPM protocol using the IoT, which mainly consists of the following four phases: (1) Network Setup Phase; (2) comparing predicted values against sensed data; (3) adding the priority level; and (4) path-loss selection. A detailed flowchart of the four phases of EERP-DPM routing protocol is shown in Figure 3.

#### 3.2.1. Network Setup Phase

Each patient should put an admitted-on medical sensor based on the recommendation of a doctor. According to the patient's health data needs, the medical personnel place the medical sensors on the patient's body. First, each patient must be registered into the Medical Server prior attaching sensors to anybody. The Aggregator initiates instructions to the network by sending control packet messages to all other sensor nodes and relays nodes about its location on the human body. The Aggregator sends a Config message to all nodes, which contains the position of Aggregator in the body; then, the position of the Aggregator gets stored. All medical sensors and relay nodes back a message, which contains sensor IDs, its position, and available residual energies in each round. In this way, all medical sensors update the Aggregator position, relays information, available residual energy, and available routes to the Aggregator. The contents of Config message are shown in Figure 4.

#### 3.2.2. Comparing Predicted Values against Sensed Data Phase

Healthcare Monitoring applications based IoT requires near real time and continuous mode data transmission to data acquisition center for a long period of time. However, in medical sensors, due to limited power resources sensing, storage and retrieval of data become critical issues, and it is difficult to perform such extensive tasks over a long period of time. Moreover, one of the most significant features of the observations collected from sensors nodes is the presence of Spatio-temporal correlation in the data, which is usually redundant. Therefore, the unnecessary transmission of these redundant data has a significant impact on reducing energy consumption.

The reduction of transmission redundant data can be achieved using the Dual Prediction Mechanism (DPM). The idea of the DPM has run the same prediction model at both the sensing nodes and the Medical server. This technique allows the sensor nodes to avoid transmitting its sensed data to the Medical server if the predictions match the collected data. In the meantime, the Medical server always presumes that its prediction reflects the real observation, unless it receives detected data from the sensor nodes. The data is transmitted if it is different from the data predicted, or data is considered critical. In this case, the critical data is transmitted to Medical server directly if it is beyond the upper/lower limits of the defined thresholds. It should be noted that the transmitting and receiving ends use the same prediction model, and they perform the same model updates for the sake of synchronization. The most essential benefit from the DPM is the ability to shrink traffic volume exchanged in the networks quite significantly. Besides, transmitting less data certainly saves sensor energy and, therefore, prolongs the lifetime of the entire network. Figures 5 and 6 illustrate the DPM work at the sensor nodes and medical server.

Sensor nodes are turned active only in their assigned time slot; else they are in sleep mode. When the sensor node gets active, it starts sensing data. Let us assume that a data memory of size *N* is used to hold the last *N* observations. At the nth time slot, the data memory is represented as *Vn* = [*Vn* − 1, *Vn* − 2, ..., *Vn* − *N*]. After that, when the Newly Detected Value (NDV) is made at time slot *n*, the information in *Vn* is used to predict the detected value. The prediction algorithm takes *Vn* as input and generates a prediction *Pn* at time slot *n*.

If the predicted value Pn was not close enough to the observed value NDV (that is, |*Pn* − NDVn| > *e*_max_, where *e*_max_ is the maximum acceptable prediction error), then the data memory will be updated as *Vn* + 1 = [NDV, *Vn* − 1,. . ., *Vn* − *N* + 1]. In this case, the prediction value and the detected value do not respect the error budget, and the sensor nodes transmit NDV to the medical server. The value NDV is used to update the prediction model variables.

However, if the predicted value *Pn* was close enough to the observed value NDV (that is, |*Pn* − ND*Vn*| ≤ *e*_max_), then *Vn* + 1 = [*Pn*, *Vn* − 1,. . ., *Vn* − *N* + 1]. Therefore, no transmission occurs because this observation can be predicted accurately. Also, the value Pn is used to update the prediction model. Meanwhile, when the medical server does not receive anything, it assumes that its prediction is within the error threshold.

#### 3.2.3. Adding the Priority Level Phase

As previously mentioned, if the predicted value *P*_*n*_ was not close enough to the observed value NDV (that is, |*Pn* − ND*Vn*| > *e*_max_), in this case, the prediction value and the detected value do not respect the error budget, and then, the sensor nodes transmit the NDV to the Medical server. For example, if the blood pressure readings suddenly exceed 180/120 mmHg, it may be signs of organ damage, and it requires immediate transmission of emergency data since the human body is suffering from severe emergency. Hence, an alert message should be sent to a doctor immediately. So, the emergency situations represent the highest priority data and should be delivered successfully to the Medical Server as soon as possible, while when the data are not critical, they are treated as a low priority packet. The direct communication is used for critical data, while multihop communication is used for normal health data delivery. After the reception of data forwarded from all the sensor nodes in a transmission round, the Aggregator aggregates the whole data into single message. This packet contains the sensor nodes IDs and their forwarded data. The pseudocode of the Added the priority level phase can be seen in Algorithm 1.

#### 3.2.4. Path-Loss Selection Phase

As previously stated, the emergency situations are the highest priority data and should be effectively delivered to the Medical Server as soon as possible. If the data are not critical, they are treated as a low priority packet. The direct communication is used for critical data, while multihop communication is used for normal health data delivery to reduce energy consumption. Furthermore, the critical sensed data is also sent quickly without any delay by utilizing the communication channel bandwidth in an efficient way. In this scheme, we have introduced two types of existing path loss models: path loss in (dB) for networking models, which represents the difference between transmitted power and received power.

In this paper, we have introduced two types of existing path loss models. The relation between the transmit and receive power is given by Friis free space equations [28, 29], which is a formula in free space that can be used for computing the Path-Loss (PL) based on the distance *d* between two communicating nodes [14]. The transmitting distance between sensor nodes and relay is denoted as *D*1, and transmitting distance between sensor nodes and the Aggregator is denoted as *D*2.

(i) If *D*1 ≤ *D*2, the sensor nodes will follow the path loss mode 1, and it is given in [14]
  (1) $$\begin{array}{c} \text{PL}\left(d,f\right)\left[dB\right]=a\times \log_{10}^{D1}+b\times \log_{10}^{f}+N_{\left(D,f\right)}. \end{array}$$
To obtain the coefficients *a*, *b*, and *N*_(*D*,*f*)_ of the approximation plane of equation (1), LMS algorithm was used. The obtained values for *a*, *b*, and *N*_(*D*,*f*)_ are −27.6, −46.5, and 157, respectively.
(ii) If *D*1 ≥ 1 *D*2, the sensor nodes will follow the path loss model 2, and it is given by
  (2) $$\begin{array}{c} \text{PL}\left(d_{i,j}\right)\left[dB\right]=PL_{0}+10n\log_{10}^{D2}+X_{\sigma },\\ {\text{PL}}_{0}=10n\log_{10}^{{\left(4\pi f\right)}^{2}/c}. \end{array}$$

## 4. Performance Analyses and Discussion

This section assesses the performance of the proposed EERP-DPM scheme from two main perspectives: first, simulation using MATLAB software; second, experimentally using the MySignals HW V2 hardware platform, which is a noticeable and comprehensive contribution from the existing work in the literature. The performance analysis of the proposed EERP-DPM scheme takes place in five indicators, namely, Network Lifetime, Residual Energy, Throughput, Path-Loss, and End-to-End Delay. This section is concluded with Table 3 that compares the proposed protocol from simulation and experimental perspectives against existing routing protocols for healthcare using the IoT.

### 4.1. Hardware Components

The vital sensing signs unit of this system is the MySignals HW V2 platform, which is a development platform for medical devices and healthcare applications.  Figure 7 represents the MySignals HW V2 platform. It monitors patients' health by deploying different medical sensors on patients' body to get sensitive data of patients for subsequent analysis by physicians. The MySignals HW V2 platform is the most complete one in the market, as it supports more than 17 biomedical sensors to measure biometric parameters such as ECG signals, blood pressure, blood oxygen, pulse, respiratory rate, and body temperature. The MySignals HW V2 platform relies on the ATmega328 microcontroller to manage various sensors and allows smart devices to communicate with it. The information gathered can be wirelessly sent using any of the 6 connectivity options available: Wi-Fi, 3G, GPRS, Bluetooth, 802.15.4, and ZigBee depending on the application. A summary of the medical sensors and the location is discussed in Table 2.

Therefore, to minimize transmitting coverage of biosensor nodes, we placed three relay nodes. The positions of these relay nodes are discussed in Table 2. In this work, we chose a low power and short-distance wireless communication module CC2540 BLE 4.0 Module made by Texas Instruments as the Relay, as Figure 8 shows. CC2540 is a highly integrated RF transceiver module for industrial use complying with Bluetooth specification V4.0 BLE. Its work spectrum locates in 2.4 GHz, which is free and is widely used in science and medical fields. This chip can ensure short-distance communication effectiveness and reliability with little components. It supports data rates as high as 250 kbps and multipoint to multipoint communication. It is characterized of small size, low cost, and low power battery [30, 31].

In contrast to the medical sensor, the Aggregator should be a device that has access to major power and resources. We have chosen a tablet that could act the Aggregator role to be a focal point between the MySignals HW V2 platform and the medical server. Therefore, the medical server is used to fill in the purpose of receiving, storing, and distributing the medical data from patients. In the proposed solution, the medical server is a PC, which has relatively powerful processing, memory, transmission capacity, and long battery life, where there is no power constraint. Further, it can be displayed in an easy-to-read format for fast assessment and action. The medical information of the patient that is stored in the medical server will be accessible by specific people who have the authorization to access such as patient himself, doctor, and patient's family member.

### 4.2. Simulation Parameters

The simulation is performed using MATLAB software to evaluate the performance and to validate the effectiveness of proposed EERP-DPM scheme. Each simulation is executed over 15,000 rounds. The simulation parameters have been indicated in Table 3. Simulation results are highlighted in Table 4.

### 4.3. Evaluation of Performance Indicators

In this subsection, we analyze the efficiency of the proposed EERP-DPM scheme in terms of five performance indicators, namely, Network Lifetime, Residual Energy, Throughput, Path-Loss, and End-to-End Delay [1, 32–35]. The rest of this subsection discusses the evaluations of these five indicators from the perspective of our proposed EERP-DPM system against two existing systems, PCRP and E-HARP, due to implantation of Dual-Prediction Mechanism and deployment of relay nodes.

#### 4.3.1. Network Lifetime

In this work, the network lifetime is defined as the total time that the nodes are alive.  Figure 9 shows simulation predictions of the proposed EERP-DPM scheme in comparison to the existing systems PCRP and E-HARP in terms of network lifetime. The average network lifetime of the EERP-DPM proposed scheme has achieved better values with average of 21,43% and 35,71%, respectively, in comparison to PCRP and E-HARP routing protocols. Clearly, the proposed EERP-DPM scheme ensures the energy-efficiency compared to the existing routing protocols. In this work, the Dual-Prediction Mechanism is used to reduce transmissions between the sensor nodes and the medical server, which has a direct impact on the network lifetime. Furthermore, the deployment of relay nodes plays a significant role to balance the energy in EERP-DPM. The better performance of the proposed EERP-DPM scheme in terms of network lifespan is due to implantation of Dual-Prediction Mechanism and deployment of relay nodes.

#### 4.3.2. Residual Energy

The node energy is always an important indicator for designing and evaluating the performance of energy-efficient routing algorithms.  Figure 10 shows predicted results from the simulation of the proposed EERP-DPM scheme in comparison to existing systems PCRP and E-HARP in terms of residual energy. As shown, we can conclude that our EERP-DPM scheme raises the residual energy beyond 51.52% and 45.5% in comparison to PCRP and E-HARP protocols, respectively. Thus, the EERP-DPM scheme conserves the energy more than PCRP and E-HARP protocols, thanks to the Dual-Prediction Mechanism. This technique allows the sensor nodes to avoid transmitting its sensed data to the medical server, as long as the predictions match the collected data, which in turn leads to a decrease in the load of the nodes and conserves the energy of sensor nodes, in addition to the deployment of relay nodes, which gives the sensor nodes more chance for direct communication via short distance. Since the relay nodes minimize the transmitting range of sensor nodes, the energy consumption of sensor nodes is reduced.

#### 4.3.3. Throughput

This performance indictor aims to measure the number of packets that can be transmitted successfully to the end medical server, where higher throughput reflects improved quality of the network. The patient monitoring system requires routing protocols that should have maximum throughput and minimum packet loss. The number of the packets received at the medical server depends on the average network life, while the average network life corresponds to the number of sensor nodes alive. The more the number of sensor nodes alive, the greater the probability of packets received at the medical server.  Figure 11 shows simulation predictions of the proposed EERP-DPM scheme in comparison to the existing systems PCRP and E-HARP in terms of throughput. The EERP-DPM protocol achieved higher throughput with average range beyond 57.62% and 27.11% in comparison to E-HARP and PCRP protocols, respectively. We can notice that the Dual-Prediction Mechanism prolongs the node's lifetime, which improves the chances of data transfer in the EERP-DPM scheme.

#### 4.3.4. Path-Loss

Path-Loss (PL) is a vital parameter for monitoring wireless system performance and network planning, which decays over distance. Basically, it is loss of power density as signals get diverted from source the destination. This term is mostly used in the wireless network for transmission of data over the network.  Figure 12 shows predicted results from the simulation of the proposed EERP-DPM scheme in comparison to existing systems PCRP and E-HARP in terms of path loss. The proposed EERP-DPM protocol shows reduced path loss with average 290 dB, which in turn reflects significant improvement in comparison to the existing data routing PCRP and E-HARP protocols.

#### 4.3.5. End-to-End Delay

End-to-End Delay is referred to as the time taken by data packet to travel from the source node to the destination node. The IoT in healthcare applications is applied for transmitting sensitive information (vital signs) from sensor nodes to the medical server. The sensed data are not always normal, where it may be critical in nature; thus, it needs to be transferred to the destination system rapidly.  Figure 13 shows simulation predictions of the proposed EERP-DPM scheme in comparison to the existing systems PCRP and E-HARP in terms of End-to-End Delay. The proposed EERP-DPM is improved by 37.14% and 40% in comparison to E-HARP and PCRP protocols, respectively. The results confirm that the EERP-DPM achieves overall minimum end-to-end delay as compared to other compared protocols, due to the presence of relay nodes on the human body, which minimizes the distance between the medical sensors and the Aggregator node.

### 4.4. Comparison between the EERP-DPM Scheme against Existing Routing Protocols

A comparison between the proposed EERP-DPM algorithm and existing routing protocols is presented in Table 4 with percentage of the increase (↑) or decrease (↓). This comparison is based on the Simulation methods, Emergency support, Network lifetime, Residual Energy, Throughput, Path-Loss, and End-to-End delay. As it can be seen, it is evident that the proposed EERP-DPM scheme of both the simulated step and experimented step satisfies most of the performance, unlike other related data routing protocols in IoT-Based Healthcare applications. In this work, the Dual-Prediction Mechanism is used to reduce transmissions between the sensor nodes and the medical server, which has a direct impact on the Evaluation of Performance Indicators. Furthermore, the deployment of relay nodes plays a significant role to balance the Performance in EERP-DPM.

Using NN fitting tool in MATLAB, the mean squared error (MSE) is measured between the proposed EERP-DPM simulated (*y*_*i*_) against experimented (*d*_*i*_) results, as per

(3) $$\begin{array}{c} \text{MSE}=\frac{1}{2}\overset{N}{\underset{j=1}{\sum }}{\left(y_{i}-d_{i}\right)}^{2}. \end{array}$$

Figure 14 shows the MSE regression plot of training, test, and validation steps, where the process determines the best number of iterations, during which validation produces a minimal value. After initial training, the process continues for 82 more iterations, during which error rates do not drop lower. During the 83 iterations, however, training stops as the error rate increases. MSE result seems reasonable since the final MSE is small; besides, there is no significant overfitting that has occurred by iteration 83, before which the best validation performance occurs.

## 5. Conclusions

The recent developments in IoT promise for providing solutions for healthcare. The medical sensors are typically equipped with batteries, which may have limited resources such as storage capacity, battery life, computational power, and channel bandwidth. Therefore, the energy-efficiency can be achieved through the development of an effective routing mechanism to prolong the network lifetime. In this paper, we propose EERP-DPM for healthcare using the IoT in order to reduce transmissions between the sensor nodes and the medical server. This technique allows the sensor nodes to avoid transmitting its sensed data to the Medical Server, as long as the predictions match the readings. The proposed system was developed and tested using a MATLAB software, and MySignals HW V2 hardware platform. We analyze the efficiency of the proposed EERP-DPM scheme in terms of five performance indicators, namely, Network Lifetime, Residual Energy, Throughput, Path-Loss, and End-to-End Delay. Both simulation and experimental results of our proposed EERP-DPM system have been evaluated from these five indicators perspective against two existing routing systems. The numerical results show that the proposed EERP-DPM protocol improves the energy utilization of the sensor nodes and prolongs the network lifetime while guaranteeing the delivery ratio besides wireless connectivity and reliability. In future, we will devise a routing protocol that considers the mobility of sensor nodes due to body movement.

## Figures and Tables

**Figure 1:** IoT-based healthcare monitoring architecture [3].

**Figure 2:** The proposed architecture of DPM-EERP solution.

**Figure 3:** Flowchart of the DPM-EERP solution.

**Figure 4:** Format of Config message.

**Figure 5:** Flowchart of the Dual-Prediction Mechanism at the Medical server.

**Figure 6:** Flowchart of the dual-prediction mechanism at the medical sensor nodes.

**Figure 7:** MySignals HW V2 platform [19].

**Figure 8:** The CC2540 platform.

**Figure 9:** Simulated results of Network Lifetime of our EERP-DPM compared to PCRP and E-HARP protocols.

**Figure 10:** Simulated results of Residual Energy of our EERP-DPM compared to PCRP and E-HARP protocols.

**Figure 11:** Simulated results of Throughput of our EERP-DPM compared to PCRP and E-HARP protocols.

**Figure 12:** Simulated results of Path Loss of our EERP-DPM compared to PCRP and E-HARP protocols.

**Figure 13:** Simulated results of End-to-End Delay of our EERP-DPM compared to PCRP and E-HARP protocols.

**Figure 14:** MSE performance of the proposed EERP-DPM simulated against experimented in MATLAB.

**Algorithm 1:** Adding the priority-level phase.

**Table 1:** A Critical Review of Routing Protocols for Healthcare using the IoT.

Protocols	Focus area(s) of the paper	Limitations
E-HARP [12]	(i) Multiattribute-based technique for dynamic cluster head (CH) selection	(i) Packet delay is high
	(ii) Cooperative routing	(ii) Network lifetime is far short
	(iii) Optimum CH is selected based on calculated cost factor (CF)	(iii) Temperature of nodes in the network is very high

PCRP [13]	(i) Emergency data will get higher priority and less delay over normal data	(i) Packets drop ratio is high
	(ii) The node with greater fitness value will be selected as a next-hop node	(ii) Network lifetime is less
	(iii) SNR parameter is used for better selection of path between sender and receiver	(iii) End-to-End delay is high

ELR-W [14]	(i) A link efficiency-oriented network model is presented considering beaconing information and network initialization process	(i) Network lifetime is less
	(ii) Path cost calculation model is derived focusing on energy aware link efficiency	(ii) High End-to-End delay

EH-RCB [15]	(i) Clustering approach to enhance nodes connectivity with each other to balance out load on single sink node	(i) Network lifetime is far short
	(ii) CF is calculated using node total energy, distance from other nodes, link SNR and required transmission power	(ii) Packet delay is high

EB-MADM [16]	(i) Dynamic cluster head selection	(i) Path loss is high
	(ii) An optimum node as cluster head which has higher residual energy level	(ii) Network lifetime is less
	(iii) Selects a new cluster head for each transmission round	
	(iv) Cooperative effort of cluster nodes	

PriNergy [17]	(i) Selecting appropriate parent member node in the RPL protocol	(i) Network lifetime is less
	(ii) Increasing network efficiency in terms of optimal speed of packet transmission in the IoT environment	(ii) Packet drop is high

EHCRP [18]	(i) Link efficiency network model is presented which calculates the capability of the forwarder node in terms of its ability to send received/sensed data	(i) Path loss is high
	(ii) Selects the forwarder node by calculating its PCE function	(ii) Network lifetime is less
		(iii) Packet drop is high

OPOT [19]	(i) Routing path is established by determining the temperature of sensor nodes to avoid hotspot region	(i) Path loss is high
	(ii) Distance between sources to destination is measured and connection is established through shortest path to minimize delay and energy consumption	(ii) Network lifetime is less
		(iii) End-to-End delay is high

Proposed EERP-DPM	(i) DPM is used to reduce transmissions between sensor nodes and the medical server	(i) Add vital computational overhead
	(ii) Data is transmitted if it is different from the data stored in previous data sensing	
	(iii) The medical server always presumes that its prediction reflects the real observation if it receives corrections from sensor nodes	
	(iv) Health data with high priority should be directly transmitted to the aggregator	

**Table 2:** Detail description of used sensors in EERP-DPM.

Node #	Sensor name	Function	Node location		Position on human body	Deployment
			*X*-axis (m)	*Y*-axis (m)		
1	EEG sensor	Measures electrical activity of muscles	0.32	1.77	Head front side	On body
2	ECG sensor	Measures electrical activity of heart	0.35	1.37	Chest (left-side)	On body
3			0.22	1.35	Chest (right-side)	On body
4	Glucose sensor	Finds blood glucose level	0.36	1.01	Stomach (left-side)	In body
5			0.35	0.01	Stomach (right-side)	In body
6	Motion sensor	Monitor the physical movement of human body	0.08	1.45	Right-side shoulder	On body
7	EMG sensor	Electrical signal is measured which is produced by human muscles	0.06	0.98	Right hand wrist	On body
8	Blood pressure sensor	Measures human body blood pressure	0.37	1.27	Left hand triceps	On body
9	Pulse oximeter sensor	Measure the amount of oxygen dissolved in blood	0.4	1.01	Left hand wrist	On body
10	Lactic acid sensor	Measure the level of lactate concentrations in blood	0.22	0.91	Right-side thigh	In body
11	Accelerometer/Gyroscope sensor	Monitor and recognize the posture movement of human body	0.45	0.45	Right-side knee	In body
12	Respiration sensor	Device used to measure the breathing rate in a patient	0.15	0.5	Left-side thigh	On body
13	Pressure sensor	Measuring the pressure through the piezoelectric effect of human tissue	0.15	0.45	Left-side lower leg	On body
14			0.25	0.17	Right-side lower leg	On body
15	Relays node 1	Multihop communication	0.3	1.03	Right-side hip	On body
16	Relays node 2		0.09	1.05	Left-side hip	On body
17	Relays node 3		0.23	1.43	Left-side thigh	On body

**Table 3:** Simulation parameters.

Parameters	Value
Number of nodes	14
*E*_trans−elect_	16.7 nJ/bit
*E*_rec−elect_	36.1 nJ/bit
*ϵ*_amp_	1.97 nJ/bit/mn
DC current (Tx)	10.5 mA
DC current (Rx)	18 mA
Supply voltage (min)	1.9 V
Packet size	4000 bits
Initial energy of sensor	0.5 J
Initial energy of relay nodes	1.0 J

**Table 4:** Qualitative comparison between EERP-DPM and other existing routing protocols.

Protocols	Performance of EERP-DPM against benchmark protocols						
	Simulator	Emergency support	Network lifetime	Residual energy	Throughput	Path-loss	End-to-end delay
E-HARP [12]	MATLAB	No	35,71% ↑	45.5% ↑	57.62% ↑	55.1% ↓	37.14% ↓
PCRP [13]	MATLAB	Yes	21,43% ↑	51.52% ↑	27.11% ↑	55.3% ↓	47.61% ↓
ELR-W [14]	NS-2	No	28.57% ↑	18% ↑	47.16% ↑	19.7% ↓	59.25% ↓
EH-RCB [15]	NS-2	No	21,43% ↑	46.54% ↑	49.15% ↑	39.44%↓	43.01% ↓
EB-MADM [16]	MATLAB	No	35,71% ↑	67,16% ↑	46.05% ↑	45.22%↓	37,71% ↓
PriNergy [17]	NS-2	Yes	21,43% ↑	24.86% ↑	25.42% ↑	11% ↓	56.25% ↓
EHCRP [18]	NS-2	No	25,71% ↑	12.83% ↑	61.01% ↓	6.3% ↓	13.39% ↓
OPOT [19]	MATLAB	No	28.57% ↑	27.86% ↑	18.98% ↑	21.3% ↓	29.23% ↓
EERP-DPM (Simulated)	MATLAB	Yes	10.37% ↑	7.68% ↑	12.31% ↑	8.78% ↓	14.36% ↓
EERP-DPM (Experimnted)	Mysignals HW V2 platform	Yes	8.77% ↑	6.36% ↑	10.98% ↑	7.3% ↓	12.43% ↓

## Data Availability

The data used to support the findings of this study are included within the article.
